# Prognostic Evaluation of CT Imaging Big Data-Assisted Arterial Chemoembolization Combined with ^125^I Seed Implantation for Non-Small-Cell Lung Cancer

**DOI:** 10.1155/2022/3472982

**Published:** 2022-07-13

**Authors:** Peng Xie, Yan Zhang, Lidong He

**Affiliations:** ^1^Sixth Medical Center of PLA General Hospital, Beijing 100048, China; ^2^China-Japan Friendship Hospital, Beijing 100048, China

## Abstract

**Objective:**

To investigate the prognostic impact of computed tomography (CT) imaging big data-assisted arterial chemoembolization combined with iodine 125 (^125^I) seed implantation on patients with non-small-cell lung cancer (NSCLC).

**Methods:**

A total of 116 patients with intermediate and advanced NSCLC hospitalized in our hospital from August 2019 to August 2020 were selected and divided into a control group and an experiment group (58 cases in each group) by random number table method for the study. The patients in the experiment group were treated with CT imaging big data-assisted arterial chemoembolization combined with ^125^I seed implantation, while the patients in the control group were treated with arterial chemoembolization alone, with the use of gemcitabine combined with cisplatin (GP) in chemotherapy. The prognostic impact was determined by analyzing recent efficacy; the incidence of adverse effects; tumor size and CT perfusion parameters including blood volume (BV), blood flow (BF), and permeability surface (PS); frailty state and quality of life; and the levels of serum tumor markers including carcinoembryonic antigen (CEA), glycoconjugate antigen 125 (CA125), cytokeratin 19 fragment antigen 21-1 (CYFRA21-1), microRNA- (miRNA-) 137, and miR-379-5p. In addition, frailty status was evaluated using the Fried frailty phenotype (FP) scale, and quality of life was determined according to Karnofsky Performance Status (KPS) score. Kaplan-Meyer (KM) method was used to analyze the survival rate of NSCLC patients after a 12-month follow-up.

**Results:**

The remission rate in the experiment group (77.59%) was higher than that in the control group (56.90%) (*P* < 0.05). Tumor size, BV, BF, PS, serum CEA and CA125 levels, and FP value in both groups were dramatically reduced after treatment compared with before treatment, especially in the experiment group after 1 and 3 months of treatment (*P* < 0.05). Meanwhile, the serum miR-137 and miR-379-5p levels and KPS scores in both groups were higher after treatment than before treatment, especially in the experiment group after 1 and 3 months of treatment (*P* < 0.05). However, there was no significant difference in the incidence of nausea and vomiting, alopecia, diarrhea, myelosuppression, and hemoptysis of NSCLC patients in both groups after treatment (*P* > 0.05). Further, the 12-month survival rate of NSCLC patients was higher in the experiment group (84.21%) than in the control group (64.29%) (*P* < 0.05).

**Conclusion:**

CT imaging big data-assisted arterial chemoembolization combined with ^125^I seed implantation for NSCLC can improve recent efficacy and the prognosis of NSCLC patients by inhibiting tumor progression with a certain degree of safety.

## 1. Introduction

Lung cancer is a malignant cancer that ranks first in mortality for both sexes among various cancers, posing a heavy burden to human health [1]. According to cancer statistics in 2015, 733,000 people were diagnosed with lung cancer, and 610,000 patients with lung cancer died in China [2]. As investigated by the American Society for Cancer Investigation (ASCI) in 2019, lung cancer ranks second in morbidity among all cancers and first in mortality among the top ten malignant cancers [3]. Non-small-cell lung cancer (NSCLC), a subtype of lung cancers, accounts for more than 80% of lung cancers [4]. Most of patients are diagnosed with NSCLC at the intermediate and advanced stage, and the opportunity for surgical treatment is missed, resulting in a poor prognosis [5].

The first-line treatment for NSCLC is chemotherapy [6]. Arterial chemoembolization has been widely used in clinical practice because of its good efficacy in treating NSCLC and advantages of less trauma and less toxic side effects compared with intravenous systemic chemotherapy [7]. In recent years, minimally invasive interventional therapy for solid tumors is developing rapidly. For example, iodine 125 (^125^I) seed implantation can accurately and continuously inhibit tumor cell proliferation, achieving the purpose of eliminating tumors [8]. Accurate surgical operation is an important guarantee for good efficacy for arterial chemoembolization and ^125^I seed implantation. A previous report indicated that computed tomography (CT) imaging data served key roles in guiding noninvasive decision support of NSCLC therapy [9]. Nevertheless, there is no data on the prognostic impact of CT imaging big data-assisted arterial chemoembolization combined with ^125^I seed implantation on NSCLC patients, which would be assessed in the present study with the hope of providing new therapeutic tactics for NSCLC.

## 2. Materials and Methods

### 2.1. NSCLC Patients and Pathological Features

A total of 116 patients with intermediate and advanced NSCLC hospitalized in our hospital from August 2019 to August 2020 were selected and divided into a control group and an experiment group (58 cases in each group) by the random number table method after obtaining approval from the Ethics Committee of our hospital. The pathological features of NSCLC patients are shown in Table 1. Tumor-node-metastasis (TNM) classification for lung cancer patients was conducted according to the reported method [10].

### 2.2. Inclusion and Exclusion Criteria for NSCLC Patients

Inclusion criteria are listed as follows: (i) patients diagnosed with NSCLC according to the diagnostic procedures [11], (ii) patients with stage III-IV NSCLC, (iii) patients undergoing initial treatment, (iv) patients whose Karnofsky Performance Status (KPS) score ≥ 70 and survival rate > 6 months, (v) patients who had no contraindications for the drugs related to the study, and (vi) patients signing the written informed consent. Exclusion criteria are as follows: (i) patients with the mental disease(s); (ii) patients with metabolic disorders like diabetes, hyperglycemia, and hyperosmolar syndromes; (iii) patients with cardiovascular and cerebrovascular diseases, liver dysfunction, and kidney dysfunction; (iv) patients diagnosed with other cancers; and (v) patients with blood system diseases and autoimmune diseases.

### 2.3. Methods

The NSCLC patients in the experiment groups were treated with CT imaging big data-assisted arterial chemoembolization combined with ^125^I seed implantation according to the following methods. Firstly, the NSCLL patients were subjected to chest CT plain scanning and enhanced chest CT scanning using an Aquilion One 320 slice CT scanner (Toshiba, Tokyo, Japan) to identify the location and scope of the lesion. Then, 5F catheter-sheath was inserted into the femoral artery by percutaneous puncture using Seldinger's technique, and 3 ~ 8 mL iohexol (320 mg/mL) was injected into the cubital vein at a rate of 1 ~ 2 mL/s to perform bronchial arteriography with puncture intubation using 5F Cobra catheter to identify the artery supplying the lesion. Afterward, the artery was administrated with 1.0 g/m^2^ gemcitabine (SFDA approval number: H20183448; Nanjing Pharmaceutical Factory, Nanjing, China) and 60~90 mg cisplatinum (CDDP; SFDA approval number: H20183341; Guangdong Lingnan Pharmaceutical Company, Guangdong, China) by puncture intubation. After 3 ~ 5 days of arterial chemoembolization, CT scanning was carried out using a radioactive particle treatment planning system (TPS) (HGGR-3000; Hokai, Zhuhai, China), and the images were transmitted to TPS to accurately delineate the tumor volume and calculate the number of ^125^I radioactive seeds, the distribution of seeds, and the layout of the puncture needles. According to the formulated individualized treatment plan provided by TPS, the implantation of ^25^I seed (1.48 × 10^7^~2.96 × 10^7^ MBp/seed; Tianjin Saide Biotechnology, Shanghai) into the edge of the central tumor was conducted using implant guns (Tianjin Saide Biotechnology). The patients in the control group were treated with arterial chemoembolization alone with the same treatment method and chemotherapy plan as the experiment group.

### 2.4. Measurement of Indexes

#### 2.4.1. Recent Efficacy

Recent efficacy was evaluated by calculating the sum of the longest diameters of target lesions according to the Response Evaluation Criteria in Solid Tumors 1.1 (RECIST 1.1) [12] after 3 months of treatment. An increase by ≥20% is considered as progression or the presence of new lesions; an increase of <20% or a decrease of <30% in the sum is considered as stability or no new appeared lesions. A reduction of ≥30% in the sum is considered a partial remission. Complete remission is considered when the target lesion is largely gone and sustained for more than 4 weeks. Remission rate was calculated according to the formula that remission rate = (complete remission + partial remission)/total number of cases × 100%.

#### 2.4.2. Tumor Size and CT Perfusion Parameters

The analysis of tumor size and CT perfusion parameters including blood volume (BV), blood flow (BF), and permeability surface (PS) was performed before treatment and after 1 and 3 months of treatment.

#### 2.4.3. Serum Tumor Markers

Venous blood was collected from NSCLC patients before treatment or after 1 and 3 months of treatment, and the serum was collected by centrifuging at 350 r/min for 5 min. Then, we analyzed the levels of carcinoembryonic antigen (CEA) and carbohydrate antigen 125 (CA125) in serum by chemiluminescence immunoassay kits (ZECEN, Taizhou, China) as per the guidebook. Serum microRNA-137 (miRNA-137) and miR-379-5p expression were quantified by quantitative real-time polymerase chain reaction (qRT-PCR) with SYBR® Premix Ex TaqTM kit (TaKaRa, Dalian, China) and analyzed by the 2^-∆∆Ct^ method.

#### 2.4.4. Frailty State and Quality of Life

Frailty state and quality of life of NSCLC patients were evaluated before treatment or after 1 and 3 months of treatment. Fried frailty phenotype (FP) scale [13] was used to evaluate frailty status, including fatigue, low physical activity, decreased grip strength, body mass, and walking speed.

### 2.5. Untoward Effects including the Incidence of Nausea and Vomiting, Alopecia, Diarrhea, Myelosuppression, and Hemoptysis

#### 2.5.1. Survival Rate

The survival rate of NSCLC patients was analyzed by Kaplan-Meyer (KM) method after a 12-month follow-up.

### 2.6. Statistical Analysis

Data were analyzed using the SPSS 22.0 software. Significant difference for attribute data was compared using *χ*^2^ test. The results of variables data were shown as means ± standard deviations. The comparisons between the two groups were performed using unpaired Student's *t*-tests or paired Student's *t*-tests. Log-rank test was used for comparing difference in Kaplan-Meier methods. *P* < 0.05 indicated statistical significance.

## 3. Results

### 3.1. Recent Efficacy

The remission rate was higher in the experiment group than in the control group after 3 months of treatment (*P* < 0.05), and the results are shown in Table 2.

### 3.2. Tumor Size and CT Perfusion Parameters

There was no difference in tumor size, BV, BF, and PS in the two groups before treatment (*P* > 0.05) (Table 3). But tumor size, BV, BF, and PS were dramatically reduced in both groups after treatment compared with before treatment, especially in the experiment group after 1 and 3 months of treatment (*P* < 0.05) (Table 3). CT images of typical cases are shown in Figures 1 and 2.

### 3.3. Serum Tumor Markers

There was no difference in serum CEA, CA125, miR-137, and miR-379-5p expression levels in the two groups before treatment (Table 4). But serum CEA and CA125 levels were dramatically reduced in both groups after treatment compared with before treatment, especially in the experiment group after 1 and 3 months of treatment (*P* < 0.05) (Table 4). Serum miR-137 and miR-379-5p expression had the opposite results (Table 4).

### 3.4. Frailty State and Quality of Life

There was no difference in FP and KPS in the two groups before treatment (Table 5). But FP was dramatically reduced in both groups after treatment compared with before treatment, especially in the experiment group after 1 and 3 months of treatment (*P* < 0.05) (Table 5). KPS had the opposite results (Table 5).

### 3.5. Untoward Effect

There was no significant difference in the incidence of nausea and vomiting, alopecia, diarrhea, myelosuppression, and hemoptysis of NSCLC patients in both groups (*P* > 0.05) (Table 6).

### 3.6. Survival Rate of NSCLC Patients

During the 12-month follow-up, one case in the experiment group was lost to follow-up (the 10th month after treatment), and 2 cases in the control group were lost to follow-up (the 7th and 9th months after treatments). The results showed that 48 patients survived and 9 cases died in the experiment group, with an 84.21% of survival rate (Figure 3(a)). In the control group, 36 patients survived and 20 cases died in the control group, with a 64.29% of survival rate (Figure 3(b)).

## 4. Discussion

CT has a high resolution for density and space and is not interfered by surrounding gas and adipose tissue, thus having great application value in NSCLC diagnosis, preoperative evaluation, and follow-up. A previous investigation has explained that valuable information about NSCLC tumor phenotypes can be acquired according to CT-based radiomic signature, thereby guiding NSCLC therapy [14].

Gemcitabine combined with cisplatin (GP chemotherapy) is required for the standard chemotherapy regimen for NSCLC [6]. Intravenous systemic chemotherapy has the disadvantage of greater systemic toxicity and side effects, leading to poor tolerance of NSCLC patients, thus causing poor chemotherapy efficacy. Compared with intravenous systemic chemotherapy, arterial chemoembolization can directly inject chemotherapy drugs into the tumor area, which can make the lesion keep high concentrations of chemotherapy drugs, thereby killing tumor cells more effectively, not affecting systemic blood concentration and liver metabolism, and helping to reduce adverse reactions [15]. The present study showed that CT imaging big data achieved good therapeutic effects in resisting arterial chemoembolization for NSCLC patients. It is because that CT scanning is helpful in puncture based on its accurate determination of the location and scope of the lesion and the artery supplying the lesion and thus ensures the accurate injection of chemotherapy drugs into the target lesion as well as the accurate killing of chemotherapy drugs to tumor cells, so as to achieve good chemotherapy effects [16]. Although arterial chemoembolization is an effective therapeutic method for NSCLC, the efficacy of chemotherapy alone is limited to a certain extent.

Radiotherapy includes external radiotherapy and internal radiotherapy, in which external radiotherapy is limited by the tolerance dose of lung tissues and its surrounding organs, resulting in a poor radiotherapy effect. Comparatively, internal radiotherapy can place radioactive substances into the lesions to achieve the purpose of precise radiotherapy and can greatly increase the dose of local radiotherapy to achieve a better radiotherapy effect. At present, the commonly used internal radiotherapy is ^125^I seed implantation. ^25^I seed implantation has been widely used to treat solid tumors, such as unresectable pancreatic cancer and NSCLC because it is almost not limited by the location and size of the lesions [17, 18]. Our data showed that the recent efficacy of CT imaging big data-assisted arterial chemoembolization combined with ^125^I seed implantation for NSCLC was higher than arterial chemoembolization alone, without significantly increasing the incidence of adverse reactions, suggesting that the combination treatment can effectively inhibit NSCLC progression. The reason for the results may be that ^125^I radioactive seeds are a kind of long half-life particles and can emit continuously low energy gamma rays, which can enhance the self-sensitization of the tumor cells and improve the sensitivity and killability of cancer cells, thus greatly improving treatment effect [19, 20].

In addition, the accurate implantation of ^125^I radioactive particles is important for therapy. CT image big data can guide the use of ^125^I radioactive particles and puncture needles and can accurately show the distribution of ^125^I radioactive seeds in the tumor after implantation, so as to ensure the therapeutic effect. Moreover, CT can measure tumor size and CT perfusion parameters [21], which can quantitatively reflect the microvessel density and blood flow velocity inside the tumor and thus is important to lung cancer therapy. In the present work, we found that CT imaging big data-assisted arterial chemoembolization combined with ^125^I seed implantation had advantages in repressing tumor growth and reducing CT perfusion parameters including BV, BF, and PS, further indicating that the combined treatment could enhance the recent efficacy of transarterial chemoembolization combined with ^125^I seed implantation. Recent data have demonstrated that serum tumor markers play key parts in evaluating the efficacy of NSCLC treatment. As reported, CEA and CA125 levels were dramatically increased in the serum of NSCLC patients but presented decreasing trends after the tumors were effectively controlled [22]. In addition, the upregulation of miR-137, a cancer-related miRNA, can inhibit cancer cell proliferation and induce cell apoptosis [23]. miR-379-5p is reduced in NSCLC tissues and cells and induces NSCLC cell proliferation inhibition and apoptosis promotion through interaction with *β*-arrestin-1, thus considered a therapeutic target for NSCLC [24]. In this work, CEA, CA125, miR-137, and miR-379-5p were employed to analyze the recent efficacy of CT imaging big data-assisted arterial chemoembolization combined with ^125^I seed implantation for NSCLC patients. The results showed that the combination therapy could decrease CEA and CA125 levels and increase miR-137 and miR-379-5p levels in the serum of NSCLC patients. Further, the combination therapy can effectively inhibit tumor progression, improve the quality of life, reduce the frailty state, and improve the survival rate of NSCLC patients. Thus, the combination therapy is a reliable method to improve the recent efficacy and long-term prognosis of NSCLC patients.

Taken together, CT imaging big data-assisted arterial chemoembolization combined with ^125^I seed implantation for NSCLC can reduce lesion blood perfusion, lesion volume, and serum CEA and CA125 levels and increase serum miR-137 and miR-379-5p levels to inhibit cancer progression, thereby improving short-term efficacy and long-term prognosis of NSCLC patients. However, a limitation should be considered when evaluating the present study. For example, the number of NSCLC patients (sample size) is small in the study, which may affect the results of the study to some extent. The limitation will be addressed in the following study.

## Figures and Tables

**Figure 1:** CT images of NSCLC patients in the control group before and after treatment. Patient Zhang XX, male, 70 years old, right lung squamous cell carcinoma, CT images before and after chemoembolization combined with 125I seed implantation. (a) Before treatment; (b) 1 month after treatment; (c) 3 months after treatment. Overall evaluation: partial relief.

**Figure 2:** CT images of NSCLC patients in the experiment group before and after treatment. Patient Zhuang XX, male, 66 years old, left lung squamous cell carcinoma, CT images before and after bronchial arterial chemoembolization. (a) Before treatment; (b) 1 month after treatment; (c) 3 months after treatment. Overall evaluation: partial relief.

**Figure 3:** Survival rate analysis of NSCLC patients after 12-month follow-up.

**Table 1:** Comparison of general information between the two groups (($\bar{x}\pm s$)/*n* (%)).

Group	*n*	Gender (male/female)	Age (year)	Body mass index (kg/m^2^)	TNM staging		Pathological typing		Cancer site		
					III period	IV period	Adenocarcinoma	Squamous carcinoma	Upper section	Middle section	Lower paragraph
Research group	58	38/20	41~76 (57.24 ± 7.52)	18.8 ~ 26.4 (23.15 ± 1.62)	37 (63.79)	21 (36.21)	42 (72.41)	16 (27.59)	12 (20.69)	27 (46.55)	19 (32.76)
Control group	58	33/25	38~75 (55.86 ± 8.10)	19.1 ~ 26.8 (23.46 ± 1.59)	40 (68.97)	18 (31.03)	45 (77.59)	13 (22.41)	10 (17.24)	31 (53.45)	17 (29.31)
*χ* ^2^/*t*		0.908	0.951	1.010	0.348		0.414			0.569	
*P*		0.341	0.344	0.301	0.555		0.520			0.753	

**Table 2:** Comparison of recent outcomes between the two groups (*n* (%)).

Group	*n*	Progress	Stable	Partial relief	Complete relief	Mitigation rate
Research group	58	3 (5.17)	10 (17.24)	31 (53.45)	14 (24.14)	45 (77.59)
Control group	58	7 (12.07)	18 (31.03)	25 (43.10)	8 (13.79)	33 (56.90)
*χ* ^2^						5.636
*P*						0.018

**Table 3:** Comparison of tumor size and CT perfusion parameters before and after treatment between the two groups ($\bar{x}\pm s$).

Time	Group	*n*	Tumor size (cm^2^)	BV (mL/100 g)	BF (mL/(min·100 g))	PS (mL/(min·100 g))
Before treatment	Research group	58	35.18 ± 5.74	9.16 ± 3.01	54.26 ± 16.85	23.50 ± 6.82
	Control group	58	33.46 ± 5.39	8.57 ± 2.82	52.07 ± 17.12	22.74 ± 6.49
	*t*		1.664	1.089	0.694	0.615
	*P*		0.099	0.278	0.489	0.540
1 month after treatment	Research group	58	25.71 ± 4.52^a^	6.15 ± 1.97^a^	28.15 ± 9.11^a^	15.43 ± 3.78^a^
	Control group	58	28.27 ± 4.86^a^	7.22 ± 2.30^a^	35.22 ± 10.35^a^	17.76 ± 4.01^a^
	*t*		2.938	2.691	3.905	3.220
	*P*		0.004	0.008	<0.001	0.002
3 months after treatment	Research group	58	19.05 ± 3.68^a^	4.47 ± 1.48^a^	19.49 ± 6.15^a^	12.95 ± 3.29^a^
	Control group	58	22.76 ± 4.07^a^	6.23 ± 1.82^a^	26.23 ± 8.17^a^	15.52 ± 3.50^a^
	*t*		5.149	5.714	5.020	4.075
	*P*		<0.001	<0.001	<0.001	<0.001

Note: compared with the same group before treatment, ^a^*P* < 0.05.

**Table 4:** Comparison of serum indexes before and after treatment between the two groups ($\bar{x}\pm s$).

Time	Group	*n*	CEA (ng/mL)	CA125 (kU/L)	miR-137	miR-379-5p
Before treatment	Research group	58	90.12 ± 15.38	75.62 ± 8.39	0.44 ± 0.08	0.40 ± 0.07
	Control group	58	88.67 ± 14.76	74.13 ± 8.21	0.46 ± 0.07	0.42 ± 0.08
	*t*		0.518	0.967	1.433	1.433
	*P*		0.605	0.336	0.155	0.155
1 month after treatment	Research group	58	42.87 ± 8.62^a^	53.16 ± 7.40^a^	0.58 ± 0.10^a^	0.55 ± 0.09^a^
	Control group	58	51.06 ± 9.54^a^	60.33 ± 8.05^a^	0.53 ± 0.08^a^	0.49 ± 0.08^a^
	*t*		4.851	4.994	2.974	3.795
	*P*		<0.001	<0.001	0.004	<0.001
3 months after treatment	Research group	58	29.17 ± 5.78^a^	44.38 ± 6.57^a^	0.63 ± 0.11^a^	0.61 ± 0.12^a^
	Control group	58	36.42 ± 6.59^a^	51.23 ± 7.18^a^	0.55 ± 0.10^a^	0.55 ± 0.10^a^
	*t*		6.299	5.360	4.098	3.925
	*P*		<0.001	<0.001	<0.001	0.004

Note: compared with the same group before treatment, ^a^*P* < 0.05.

**Table 5:** Comparison of debilitating status and quality of survival before and after treatment between the two groups ($\bar{x}\pm s$, points).

Time	Group	*n*	FP	KPS
Before treatment	Research group	58	4.05 ± 0.68	78.39 ± 4.56
	Control group	58	4.01 ± 0.65	79.12 ± 5.10
	*t*		0.234	0.813
	*P*		0.747	0.418
1 month after treatment	Research group	58	3.18 ± 0.50^a^	85.21 ± 4.73^a^
	Control group	58	3.49 ± 0.53^a^	82.54 ± 4.60^a^
	*t*		3.240	3.082
	*P*		0.002	0.003
3 months after treatment	Research group	58	2.09 ± 0.42^a^	89.74 ± 5.12^a^
	Control group	58	2.45 ± 0.47^a^	86.31 ± 4.89^a^
	*t*		4.350	3.690
	*P*		<0.001	<0.001

Note: compared with the same group before treatment, ^a^*P* < 0.05.

**Table 6:** Comparison of the occurrence of adverse reactions between the two groups (*n* (%)).

Group	*n*	Nausea and vomiting	Hair loss	Diarrhea	Bone marrow suppression	Hemoptysis
Research group	58	26 (44.83)	15 (25.86)	9 (15.52)	22 (37.93)	17 (29.31)
Control group	58	21 (36.21)	11 (18.97)	6 (10.34)	19 (32.76)	10 (17.24)
*χ* ^2^		0.894	0.793	0.689	0.340	2.365
*P*		0.344	0.373	0.407	0.560	0.124

## Data Availability

The labeled dataset used to support the findings of this study are available from the corresponding author upon request.
